The article "miRNA-221 Regulates Spinal Cord Injury-Induced Inflammatory Response through Targeting TNF-α Expression" was retracted in 2024. Reasons: signs of a paper mill; a false affiliation; unreliable results or conclusions.

# miRNA-221 Regulates Spinal Cord Injury-Induced Inflammatory Response through Targeting TNF-*α* Expression

**DOI:** 10.1155/2021/6687963

**Published:** 2021-04-07

**Authors:** Feng Sun, Haiwei Zhang, Tianwen Huang, Jianhui Shi, Tianli Wei, Yansong Wang

**Affiliations:** ^1^Department of Spine Surgery, The First Affiliated Hospital of Harbin Medical University, Harbin, 150001 Heilongjiang Province, China; ^2^Department of Orthopaedic Surgery, General Hospital of General Administration of Agriculture and Reclamation, Harbin, Heilongjiang Province 150088, China; ^3^Department of Imaging, General Hospital of General Administration of Agriculture and Reclamation, Harbin, Heilongjiang Province 150088, China; ^4^Department of Orthopaedics, Heilongjiang Provincial Hospital, No. 82, Zhongshan Road, Harbin, Heilongjiang Province 150036, China

## Abstract

**Objectives:**

To investigate the roles of miR-221 in spinal cord injury (SCI) as well as the underlying mechanism.

**Methods:**

A mouse model of SCI was generated and used to examine dynamic changes in grip strength of the mouse upper and lower limbs. The expression of miR-221 and tumor necrosis factor-*α* (TNF-*α*) was detected by RT-qPCR and Western blot. Levels of inflammation and oxidative stress in microglia cells of the injured mice overexpressing miR-221 were then measured by ELISA. Bioinformatics analysis and dual-luciferase reporter assay were conducted to identify the miR-221 target.

**Results:**

We successfully constructed SCI mouse model. The results of qRT-PCR showed that miR-221 was gradually upregulated in the spinal cord tissue of mice in the SCI group with the prolonged injury time. At the same time, the mRNA and protein of TNF-*α* gradually decreased. We further confirmed through cell experiments that the inflammatory factors TNF-*α* and IL-6, as well as iNOS and eROS, were upregulated in spinal cord microglia cells of SCI mice, and upregulation of miR-122 can inhibit their expression. Finally, the luciferase reporter experiment confirmed that miR-122 targeted TNF-*α*.

**Conclusions:**

We present evidence that miR-221 promotes functional recovery of the injured spinal cord through targeting TNF-*α*, while alleviating inflammatory response and oxidative stress.

## 1. Backgrounds

Spinal cord injury (SCI) refers to an injury to the spinal cord resulting from direct or indirect external forces [1]. The morbidity of the disease has been rising yearly. It has been reported that while there are 11,000 new SCI patients in the United States, the number of the new cases in China can be as high as 60,000 [2]. It was widely believed that the spinal cord has a poor ability to self-repair the injury. However, scientists found that under the right conditions, the spinal cord is capable of regenerating nerve cells, making it possible for the spinal cord to recover from injury [3]. A growing number of studies demonstrate that immune inflammatory response following SCI plays a vital role in the process of injury and recovery [4, 5]. To date, roles of the inflammatory response in the indicated process have been validated in the animal models [6].

The article "miRNA-221 Regulates Spinal Cord Injury-Induced Inflammatory Response through Targeting TNF-α Expression" was retracted in 2024. Reasons: signs of a paper mill; a false affiliation; unreliable results or conclusions.

Recent studies have shown that microRNAs (miRNAs) significantly regulate the secondary injury to SCI as well as neural regeneration process following the injury. Thus, studies on SCI-related miRNAs could improve the understanding of disease progression, thereby facilitating the treatment and prognostic prediction of SCI [7, 8]. miRNAs are a class of noncoding small RNA molecules consisting of approximately 22 nucleotides, which regulate transcriptional expression of the target genes. As transcriptional regulators, miRNAs are capable of regulating protein synthesis, thus being involved in every stage of disease and development [9]. miRNAs act in regulating the development and functional perfection of the nervous system under physiological conditions, including the maintenance of normal morphological structure of nerve cells, axon growth, synaptic plasticity, function, and morphological maintenance [10]. In the meantime, miRNAs have been shown to be involved in SCI processes under pathological conditions and to reflect the severity of injuries to a certain extent [11]. miRNAs may participate in the nerve degeneration, and prompting the miRNA expression changes may also be involved, including spinal cord trauma after secondary [12] and the central nervous system damage. Yunta et al. reported that SCI traumatic SD rat model was constructed, and the expression of miRNAs in rats at different time points after SCI, bioinformatics analysis results show that the changes on the expression of microRNAs involved including inflammatory reaction, cell apoptosis, and astrocyte proliferation multiple SCI pathophysiological process of [13, 14].

An RNA-SEQ technology-based analysis of the expression profiles of miRNAs and mRNAs in SCI patients identified significant changes in miR-221 expression. Based on this observation, we used SCI animal model and the transfected cells to preliminarily explore the mechanism underlying the regulatory role of miRNAs in SCI process. This study may provide theoretical basis for developing targeted therapy of SCI.

## 2. Materials and Methods

### 2.1. Animal and Reagents

60 clean-grade healthy C57BL/6 male adult mice (28-30 g, 3 months) were provided by Beijing Viton Lever Animal Experiment Center (certificate No. SCXK (Beijing) 2006-0009). Mice were fed with standard diet, had free access to water, and reared at 22~24°C and 55%~60% humidity and normal day-night alternations. The reagents were purchased as follows: TRIzol Reagent from Invitrogen, USA; miR-221 agonist Agomir-221 and negative control Agomir-NC from Guangzhou Ruibo Biotechnology Co., LTD; PrimeScript RT Reagent Kit with gDNA Eraser and Fluorescent quantitative PCR kit (SYBR Premix Ex Taq TM) from TaKaRa, Japan; IL-1, TNF-*α*, and Caspase-3 rabbit anti-mouse polyclonal antibodies from Abcam, USA; GAPDH rabbit anti-mouse polyclonal antibody and horseradish peroxidase-labeled sheep anti-rabbit IgG from Wuhan Baidu Biotechnology Co., LTD; and In Situ Terminal Labeling (TUNEL) assay kit and LightCycler PCR instrument from Roche, USA. All primers were designed and synthesized by Shanghai Jikeiyin Chemical Technology Co., LTD.

The article "miRNA-221 Regulates Spinal Cord Injury-Induced Inflammatory Response through Targeting TNF-α Expression" was retracted in 2024. Reasons: signs of a paper mill; a false affiliation; unreliable results or conclusions.

### 2.2. Establishment of C5 Spinal Cord Contusion Model

The SCI group was dissected longitudinally to expose the C4-6 spinous process. The C5 lamina was then removed, exposing the dural sac and damaging the C5 spinal cord. Once the wound is successful, the bleeding was stopped, and the incisions in muscle, fascia, and skin were closed. The dural sac is also exposed. Protective measures were taken to prevent damage to the dural sac and spinal cord.

### 2.3. Measurement of Forearm Grip Strength

Four successful grip strength measurements were recorded, and the mean values were recorded. If the forelimb movement disorder is too severe for the mice to grasp the bar, the score of grip strength is 0. The front limb movement scale (FLS) was measured, and the mice were recorded in a 90 × 120 cm wide field of vision and observed for 4 minutes. FLS scores were recorded by the two subjects and ranged from 0 to 17 based on severity.

### 2.4. Hematoxylin-Eosin (HE) Staining

The mice were sacrificed, and the spinal cord tissues were isolated. The tissues were then fixed with 4% paraformaldehyde at 4°C for 48 h. Subsequently, the tissues were embedded in paraffin, sectioned, and stained in strict accordance with the manufacturer's instructions of the HE staining kit.

### 2.5. Cell Culture and Treatment

Mouse spinal cord tissue from each group was removed and cultured in mixed cell culture medium for 2 days. Next, DMEM medium (Kengan, Nanjing, China) containing 20% FBS was substituted for the Eagle medium. Microglia cells were then isolated after 10 days.

### 2.6. Quantitative Real-Time PCR (qRT-PCR)

The mRNA levels of mouse spinal cord tissue and transfected cells with miR-NC or miR-221 mimic were determined using qRT-PCR. TRIzol reagents were used to extract total RNA of tissue or transfected cells. qRT-PCR was carried out using PrimeScript reverse transcription kit and SYBR Premix, and the expression of GAPDH was used for internal normalization.

The article "miRNA-221 Regulates Spinal Cord Injury-Induced Inflammatory Response through Targeting TNF-α Expression" was retracted in 2024. Reasons: signs of a paper mill; a false affiliation; unreliable results or conclusions.

### 2.7. Western Blotting

After 48 h of transfection, the cells and damaged tissues were collected and the total protein was extracted by radioimmunoprecipitation (RIPA). Total protein was separated through 10% SDS-PAGE and then transferred to PVDF. The membranes were blocked with 5% skimmed milk and were incubated with primary antibodies TNF-*α*, induced nitric oxide synthase (iNOS), or endothelial nitric oxide synthase (eROS) (American expression vector, Carlsbad, CA) at 4°C overnight, followed by horseradish peroxidase (us) rabbit immunoglobulin (American expression vector, Carlsbad, CA). The protein bands were exposed by chromogenic agents, and the protein expression was analyzed by the gene tool software.

### 2.8. Double Luciferase Reporter Assay

TNF-*α* 3′-UTR was inserted into the vector for transformation. 150 ng of the extracted plasmid was mixed with 3 pmol miR-221 mimics or mimic NC and then added into Opti-MEM medium containing 1 Lipofectamine. The mixture was subsequently subjected to 30 min of incubation at room temperature. Thereafter, it was added to the corresponding microglia cells and incubated for 24 hours. Double luciferase assay was performed according to the method of Copoeia (Rockville, MD, USA).

### 2.9. Enzyme-Linked Immunosorbent Assay (ELISA)

The levels of TNF-*α* and IL-10 in the supernatants of lysed cells were determined by using an ELISA kit (Boster, Wuhan, China). OD values at the wavelength of 450 nm were recorded, and the standard curve was used to quantify the expression of TNF-*α* and IL-10.

### 2.10. Statistics Analysis

All data are reported as means ± standard deviation (SD). Statistical analysis was carried out by using the SPSS 17.0 software (SPSS Inc., Chicago, IL, USA). A one-way analysis of variance (ANOVA) followed by LSD test was used for multiple comparisons among different groups. *p* < 0.05 indicates statistical significance.

## 3. Results

### 3.1. SCI Mouse Model Was Successfully Established

In order to confirm whether the SCI model is successful, we tested the grip strength of the mouse forelimbs. The results (Figure 1(a)) showed that the early grip recovery of the SCI group was significantly slower than that of the sham operation group. One month after the operation, the grip strength of the mice in the sham operation group gradually returned to normal. In contrast, the injured mice in the SCI group were unable to do any movement of their front paws after the operation. During 21 d-52 d, the gripping power of the two claws gradually increased over time. It was worth noting that, compared with the sham operation group, the grip strength of the SCI group was significantly reduced at all time points after surgery. Furthermore, we detected the pathomorphological changes of the spinal cord tissue of the two groups of mice by HE staining. There was no obvious damage to the spinal cord tissue structure in the sham operation group. In the SCI group, the spinal cord tissue structure is disordered, the gray matter area was destroyed and dissolved, and the necrotic area was larger (Figure 1(b)).

The article "miRNA-221 Regulates Spinal Cord Injury-Induced Inflammatory Response through Targeting TNF-α Expression" was retracted in 2024. Reasons: signs of a paper mill; a false affiliation; unreliable results or conclusions.

### 3.2. Increased Expression of miR-221 and Reduced Expression of TNF-*α* in Injured Spinal Cords

The qRT-PCR assay revealed a stepwise increase in miR-221 expression within 7 days following injury. To validate this finding, we assessed miR-221 and TNF-*α* expression. In the experiments, miR-221 expression in mouse spinal cord of the sham group on the first day after surgery was used as a control. The results showed that while miR-221 expression in the injury group was increased gradually, a time-dependent decrease in TNF-*α* expression was evident (Figures 2(a)–2(d)). These results showed that miR-221 and TNF-*α* participated in the occurrence and development of SCI.

### 3.3. miR-221 Regulates Inflammation following Spinal Cord Injury

Next, ELISA was performed to analyze the alterations in the expression of cytokines induced by miR-221 during SCI. We observed that the expression of inflammatory cytokines TNF-*α* and IL-6 was significantly increased in the damaged mouse glial cells, but overexpression of miR-221 could decrease the expression of TNF-*α* and IL-6 (Figure 3(a)). Meanwhile, overexpression of miR-221 could significantly downregulate the increased expression of iNOS and eROS in the injured mice (Figure 3(b)). These results suggested that miR-221 could inhibit inflammatory response, reduce oxidative stress, and significantly alleviate SCI.

### 3.4. miR-221 Targets TNF-*α* to Regulate Inflammatory Responses after Spinal Cord Injury

Bioinformatics analysis revealed that TNF-*α* is a potential miR-221 target. We then undertook a dual-luciferase reporter assay to investigate if TNF-*α* has a binding site of miR-221. The assay demonstrated that miR-221 markedly downregulated the luciferase activities in wild-type TNF-*α* scorpion cells, but not in the mutant cells. Moreover, the overexpression of miR-221 resulted in significantly reduced TNF-*α* expression at both mRNA and protein levels. Taken together, these data indicate that TNF-*α* is a downstream target of miR-221, while suggesting that miR-221 can alleviate spinal cord injury-induced inflammatory response and oxidative stress through targeting TNF-*α*, thereby facilitating the spinal cord recovery (Figures 4(a) and 4(b)).

The article "miRNA-221 Regulates Spinal Cord Injury-Induced Inflammatory Response through Targeting TNF-α Expression" was retracted in 2024. Reasons: signs of a paper mill; a false affiliation; unreliable results or conclusions.

## 4. Discussion

SCI is a serious central nervous system disease that can cause severe leg dysfunction and even paralysis for life [15]. In recent years, the important regulatory role of miRNA in the pathological process of SCI has also been gradually confirmed. Studies have shown that miRNAs are essential in regulating inflammation signaling pathways and pathological immune responses [16]. To date, many miRNAs have been identified to be differentially expressed in the central nerve system, including mouse spinal cord [17–19]. miRNAs act in regulating the expression of various transcription factors critically involved in the development and functional establishment of the spinal cord, including neuronal cell differentiation and cell type maintenance. It has been reported that IL-7-induced inflammation can effectively downregulate miR-136-5p expression [20]. Notably, miR-99b-5p regulates spinal nerve injury in mice through the mTOR pathway [21], while miR-214-3p and miR-211 are critically involved in the repair of injured spinal cord [22, 23]. Therefore, functional study of miRNAs in spinal cord injury could provide evidence for future treatment.

For this purpose, we first established a SCI model. The experimental animal model is a modified C5 spinal cord contusion model. The establishment of animal models in this study is similar to human spinal cord injury [24] and then tested grip strength recovery of the mouse upper and lower limbs. Strikingly, the upper and lower limb strength recovery can be detected as early as 7 days postinjury. Next, we found that miR-221 expression was increased in a time-dependent manner during SCI. Meanwhile, we observed that TNF-*α* expression decreased over time. These results confirmed that miR-221 and TNF-*α* played important roles in the occurrence and development of SCI.

We subsequently measured the levels of inflammation and oxidative stress in the injured mouse model and found that inflammatory markers (TNF-*α* and IL-6) and oxidative stress index (iNOS and eROS) were significantly upregulated. However, overexpression of miR-221 could significantly inhibit the expression of these factors. This is similar to the results of the DAI study; miR-137 can attenuate SCI by inhibiting NEUROD4 through reducing inflammation and oxidative stress [7].

Finally, while bioinformatics analysis predicted TNF-*α* as a potential miR-221 target, the dual-luciferase assay demonstrated that TNF-*α* was expressed with miR-221, and miR-221 overexpression caused significantly reduced expression of TNF-*α*. Overall, the findings in this study led us to propose that miR-221 downregulates TNF-*α*, a rehabilitation target of spinal cord injury, while inhibiting inflammatory response and oxidative stress in the injured mice.

The article "miRNA-221 Regulates Spinal Cord Injury-Induced Inflammatory Response through Targeting TNF-α Expression" was retracted in 2024. Reasons: signs of a paper mill; a false affiliation; unreliable results or conclusions.

## Figures and Tables

**Figure 1:** SCI mouse model was successfully established. (a) Grip strength of mice in the pair forepaws. (b) Observation of morphology of spinal cord tissues in the sham and SCI group detected by HE staining.

**Figure 2:** Dynamic changes of miR-221 and TNF-*α* expression. (a) A significant time-dependent increase in miR-221 expression during the injury. (b–d) The time-dependent decrease in TNF-*α* expression.

**Figure 3:** miR-221 downregulates the levels of inflammatory cytokines and oxidative stress. (a) miR-221 inhibited the expression of TNF-*α* and IL-6. (b) miR-221 markedly alleviated oxidative stress. ^∗∗^*p* < 0.01 vs. sham group; ^##^*p* < 0.01 vs. SCI+NC group.

**Figure 4:** TNF-*α* was a direct target gene of miR-221. (a) The binding sequence of TNF-*α* and miR-221. (b) Luciferase report assay demonstrated that miR-221 overexpression suppressed the luciferase activity of wild-type (WT) 3′-UTR of TNF-*α*. ^∗^*p* < 0.05.

## Data Availability

Some or all data, models, or code generated or used during the study are available from the corresponding author by request.
